The article "The Clinical Efficacy of Clopidogrel Bisulfate Tablets Combined with Olmesartan Medoxomil for Ischemic Stroke with Hypertension and the Effect of Angiotensin II Type 1 Receptor Level on Prognosis" was published in 2021. Journal: Comput Math Methods Med.

# The Clinical Efficacy of Clopidogrel Bisulfate Tablets Combined with Olmesartan Medoxomil for Ischemic Stroke with Hypertension and the Effect of Angiotensin II Type 1 Receptor Level on Prognosis

**DOI:** 10.1155/2021/4487393

**Published:** 2021-10-27

**Authors:** Jia Yu, Wei Fang, Xing Guo, Haiyang Jiang, Peng Sun, Yufeng Liu, Xin Jin

**Affiliations:** ^1^Department of Neurosurgery, Tangdu Hospital, Air Force Military Medical University, Xi'an, 710038, China; ^2^Department of Nursing, Tangdu Hospital, Air Force Military Medical University, Xi'an, 710038, China

## Abstract

**Background:**

Ischemic stroke combined with hypertension can increase risks of stroke recurrence and death.

**Aim:**

The aim of this study is to investigate the clinical efficacy of clopidogrel bisulfate tablets combined with olmesartan medoxomil in the treatment of ischemic stroke patients with hypertension and the effect of angiotensin II type 1 receptor (AT_1_R) level on prognosis.

**Methods:**

Ninety ischemic stroke patients with hypertension were chosen for continuous treatment with clopidogrel bisulfate tablets and olmesartan medoxomil for 12 months. The Modified Edinburgh Scandinavian Stroke Scale (MESSS) score, Brunnstrom score, Barthel score, death, recurrence, and progression of cerebrovascular residual lesions were observed and recorded during the treatment period. According to the plasma AT_1_R expression of the patients before treatment, the patients were divided into a high-AT_1_R group and low-AT_1_R group. Then, survival analysis was performed.

**Results:**

Compared with pretreatment, the MESSS scores of the patients at the first, second, third, sixth, ninth, and twelfth months after treatment were reduced (*p* < 0.01) while the Brunnstrom score and Barthel score were prominently boosted (*p* < 0.01). Compared with the low-AT_1_R group, patients in the high-AT_1_R group had higher rates of stroke recurrence and progression of residual cerebrovascular lesions (*p* < 0.05).

**Conclusion:**

Clopidogrel bisulfate tablets combined with olmesartan medoxomil has prominent clinical effects in the treatment of ischemic stroke patients with hypertension, evidently improving the prognosis. In addition, the level of AT_1_R may be a vital factor affecting the prognosis.

## 1. Introduction

Stroke is one of the leading causes of death and disability worldwide, which brings a heavy economic burden to the healthcare system [1]. All over the world, one in six people may suffer a stroke in their lifetime, and more than 13.7 million cases occur each year [2]. Ischemic stroke accounts for 71% of all stroke cases [3]. Comorbidity, a sign of ischemic stroke, will accelerate the incidence of ischemic stroke and affect the prognosis [4, 5]. Unlike pediatric stroke, the main comorbidities of adult ischemic stroke are hypertension, diabetes, hyperlipidemia, and/or changes in coagulation status (such as pregnancy and preeclampsia) [6]. Among them, hypertension is very common in people with ischemic stroke and is the most important risk factor for ischemic stroke [6, 7]. Studies proved that antihypertensive therapy reduces the incidence of ischemic stroke, and a decrease of 5-6 mmHg in systolic blood pressure and/or a 2-3 mmHg decrease in diastolic blood pressure can reduce the relative risk of stroke by 40% [8, 9]. Hence, the control of hypertension is extremely crucial for patients with ischemic stroke. For the past few years, with the development of medical technology, there have been a lot of studies on the treatment of single disease of ischemic stroke and hypertension, and remarkable progress has been achieved [10, 11]. However, few studies have evaluated the efficacy and prognosis of targeted treatments for ischemic stroke combined with hypertension.

Angiotensin (Ang) plays a vital role in blood pressure regulation and participates in the development of diseases such as hypertension, stroke, cerebral aneurysm, atherosclerosis, and heart failure [12, 13]. Ang II type 1 receptor blockers (ARB) have a beneficial effect on preventing the recurrence of stroke [14]. Ang II-mediated blood pressure regulation is achieved by binding to angiotensin II type 1 receptor (AT_1_R) [15]. Compared with other ARBs, olmesartan has a higher binding level with AT_1_R and has a stronger antihypertensive effect [16]. As a result, in this study, olmesartan medoxomil was utilized for blood pressure-lowering treatment in patients with ischemic stroke and hypertension.

Antiplatelet aggregation is currently the primary treatment for ischemic stroke [17]. Aspirin is the first antiplatelet aggregation treatment drug. Antihypertensive drugs combined with aspirin are often applied in clinical as the first choice for the secondary prevention of ischemic stroke and hypertension [18]. However, long-term use of aspirin increases the risk of bleeding and 10% of patients have drug resistance, which makes aspirin not widely utilized in clinical practice [19, 20]. Hence, how to combine antihypertensive drugs and antiplatelet aggregation drugs to treat ischemic stroke combined with hypertension to improve the prognosis has become one of the crucial research topics for clinicians.

According to reports, one of the metabolites of clopidogrel is a platelet aggregation inhibitor, which selectively represses the binding of adenosine diphosphate (ADP) to its platelet P2Y12 receptor and suppresses the secondary ADP-mediated activation of the glycoprotein GPIIb/IIIa complex [21]. A study proved that the inhibitory effect of clopidogrel on platelet function can decrease the risk of ischemic stroke [22]. As a result, this study applied clopidogrel bisulfate tablets combined with olmesartan medoxomil in the treatment of ischemic stroke patients with hypertension, aiming at investigating the clinical effects of the combination therapy and related factors affecting the prognosis.

## 2. Information and Methods

### 2.1. General Information

Ninety patients with a history of hypertension who were admitted to the Department of Neurology of Tangdu Hospital, Air Force Military Medical University, from March 2019 to March 2021 and confirmed by magnetic resonance imaging (MRI) or computed tomography (CT) as a new-onset ischemic stroke were selected for research. Among them, 52 were males and 38 were females, with an average age of (65.31 ± 7.56) years, and the average time from onset to admission was 24.51 ± 4.09 h. The study protocol was approved by the hospital medical ethics committee of Tang Du Hospital, Fourth Military Medical University (TDLL-KY-202107-02), and the informed consent forms were in writing signed by the patients or their family members.

### 2.2. Inclusion Criteria

The inclusion criteria are as follows: (1) comply with the diagnosis of patients with hypertension and ischemic stroke in the “Guidelines for Prevention and Treatment of Hypertension in China” [23] and “Guidelines for Prevention and Treatment of Cerebrovascular Diseases in China” [24]; (2) onset time ≤ 7 d; (3) no allergic reaction to the drugs used in this study; and (4) clear consciousness.

### 2.3. Exclusion Criteria

The exclusion criteria are as follows: (1) patients with cardiogenic embolism, low left ventricular ejection fraction, and severe arrhythmia; (2) patients with intracerebral hemorrhage; (3) patients with severe liver and kidney disease; (4) patients taking drugs that affect this study 7 d before treatment; and (5) patients having poor compliance without taking medication regularly after discharge. The flow chart of screening patients is shown in Figure 1.

### 2.4. Treatment Methods

After the patients were admitted to the hospital, they received oral clopidogrel bisulfate tablets (CSPC PHARMA Ouyi Pharmaceutical Co., Ltd., SFDA approval number H20193160) on the basis of routine basic treatment, 75 mg each time, once a day. At the same time, the patients were given olmesartan medoxomil (Daiichi Sankyo Pharmaceutical (Shanghai) Co., Ltd., H2018009), with an initial dose of 20 mg, once a day. For patients whose blood pressure was higher than 140/90 mmHg after 2 weeks of treatment, the dose was increased to 40 mg.

### 2.5. Observation Indicators and Follow-Up

Before treatment, MESSS score [25], Brunnstrom hemiplegia function evaluation [26], and Barthel index score [27] were performed. The progression of residual cerebral vascular foci, recurrent stroke, and death was recorded according to the diagnostic criteria in the guidelines [24]. Patients were followed up once a month during the first 3 months after treatment. Follow-up was performed every 3 months until 12 months after treatment.

### 2.6. Detection of AT_1_R Level in Plasma

The plasma in the heparin anticoagulation tube of the patient was collected before treatment, and the enzyme-linked immunosorbent assay (ELISA) was applied. The kit was acquired from ADL, USA, and the microplate reader model was Clinibio-128C. The ELISA plate was taken out, and the standard holes and sample holes were numbered in sequence. Firstly, 100 *μ*L of standard preparations was added to each well; 50 *μ*L of enzyme labeling solution was added to the standard and sample holes and incubated at 36 ± 2°C for 1 h. Each well was washed 5 times with a plate washer, and let it stand for 10-20 s each time. Then, 50 *μ*L of A and B solution was added to each well and incubated at 36 ± 2°C in the dark for 15 min. Next, 50 *μ*L stop buffer was added to each well to stop the reaction. Negative and positive controls were set up in the reaction. After the reaction was completed, the absorbance value of each well was read on a microplate reader at a wavelength of 450 nm. A standard curve was plotted according to the standard preparations, and the relative expression level of AT_1_R of each specimen was calculated.

### 2.7. Statistical Methods

All data in this study were analyzed using SPSS 22.0 statistical software. A paired *t*-test was utilized for comparison before and after drug treatment. The Kaplan-Meier method was applied for the analysis of progression-free survival. Log-rank test was employed to compare survival between groups to compare the progression-free survival rate, recurrence-free survival rate, and overall survival rate of cerebrovascular residual lesions between the high- and low-level AT_1_R groups from pretreatment to 12 months after treatment. *p* < 0.05 was considered statistically significant.

## 3. Results

### 3.1. Baseline Characteristics

Following the inclusion and exclusion criteria, 90 patients diagnosed with ischemic stroke and hypertension in Tangdu Hospital, Air Force Military Medical University, were included in the study. The baseline characteristics are listed in Table 1. The average age of the patients was 63.96 ± 6.10 years, including 52 males and 38 females. The average systolic blood pressure of the patients on admission was 162.02 ± 10.14 mmHg, and the diastolic blood pressure was 93.12 ± 7.57 mmHg.

### 3.2. Comparison of MESSS Scores before and after Treatment

To evaluate the efficacy of clopidogrel bisulfate tablets combined with olmesartan medoxomil in the recovery of patients' neurological function, the MESSS score was performed in this study. A total score of ≤15 points was considered as mild neurological deficit, ≤30 points as moderate neurological deficit, and ≥31 points as severe neurological deficit. Higher score indicated more severe neurological deficit. The results revealed that compared with before treatment, the MESSS scores of patients at 1 month, 2 months, 3 months, 6 months, 9 months, and 12 months after treatment were evidently reduced (Table 2, *p* < 0.01).

### 3.3. Comparison of Brunnstrom Score before and after Treatment

In an effort to evaluate the effect of clopidogrel bisulfate tablets combined with olmesartan medoxomil treatment on the recovery of hemiplegic motor function in patients with ischemic stroke and hypertension, patients with hemiplegic motor function were divided into 1-6 grades following Brunnstrom staging. Level 1 was the paralysis period, level 2 was the joint reaction period, level 3 was the joint exercise period, level 4 was the separation exercise out of the common movement mode, level 5 was the further improvement of the separation exercise, and level 6 was the coordinated movement and roughly normal movement speed. As revealed by the results, compared with the Brunnstrom score before treatment, the Brunnstrom score of patients at 1, 2, 3, 6, 9, and 12 months after treatment was markedly improved, and the motor function of hemiplegic limbs was prominently restored (Table 3, *p* < 0.01).

### 3.4. Comparison of Activities of Daily Living before and after Treatment

In this study, the modified Barthel index score was applied to evaluate the recovery of activities of daily living in ischemic stroke patients with hypertension after clopidogrel bisulfate tablets combined with olmesartan medoxomil. The higher the score was, the stronger the patient's ability to perform activities of daily living was. As indicated in the results, the patients' activities of daily living at 1 month, 2 months, 3 months, 6 months, 9 months, and 12 months after treatment were evidently improved than before treatment (Table 4, *p* < 0.01).

### 3.5. The Effect of the Expression Level of AT_1_R on the Progression of Cerebrovascular Residual Lesions

Olmesartan is a selective AT_1_R antagonist, which blocks the vasoconstrictive effect of AT_1_R by selectively blocking the binding of AT_1_R and vascular smooth muscle AT_1_R. In an effort to explore whether AT_1_R level affects the prognosis of ischemic stroke patients with hypertension, this study divided patients into a high-AT_1_R group and low-AT_1_R group based on their plasma AT_1_R level before treatment. Then, differences in the progression, recurrence, and overall survival time of the residual cerebrovascular lesions between the two groups were evaluated by progression-free survival analysis. It was revealed that compared with patients with low AT_1_R, patients with high AT_1_R had a higher risk of progression in the sequelae period of residual cerebrovascular lesions (Figure 2, *p* = 0.029).

### 3.6. The Effect of AT_1_R Expression Level on the Recurrence of Stroke

To evaluate the effect of the expression level of AT_1_R on the recurrence of stroke in patients with ischemic stroke, we conducted a 12-month follow-up on the recurrence of patients. The results suggested that compared with the low-AT_1_R group, the stroke recurrence rate was higher in the high-AT_1_R group, and the difference was statistically significant (Figure 3, *p* = 0.016).

### 3.7. The Expression Level of AT_1_R and Its Effect on Survival Time

Within 12 months after treatment, there were 2 deaths (4.44%, 2/45) in the high-AT_1_R group and 1 death (2.22%, 1/45) in the low-AT_1_R group. There was no statistically significant difference in overall survival between the two groups (Figure 4, *p* = 0.541).

## 4. Discussion

Ischemic stroke often occurs in people around 55 years of age. It has the characteristics of rapid progress, poor prognosis, and high disability rate. In the early stage, it may cause brain tissue necrosis, softening, ischemia, and hypoxia due to the occlusion and reduction of local blood supply of brain tissue. The main manifestations are declines of sensory function, visual function, language function, and motor function, which seriously affect the patient's daily life. If the treatment is not timely, it can also endanger life and safety and aggravate neurological damage [28, 29].

Currently, antiplatelet aggregation drugs are often used in clinical to treat ischemic stroke. Antiplatelet aggregation drugs can effectively reduce the mortality rate of ischemic stroke and the recurrence rate of early ischemic stroke and reduce the cardiac complications caused by cerebral infarction. One of the representative drugs is clopidogrel bisulfate [21, 30]. The study of Rahman et al. [31] uncovered that compared with aspirin monotherapy, aspirin plus clopidogrel treatment can evidently reduce the risk of ischemic stroke recurrence and prominently reduce the occurrence of adverse cardiovascular events, which is consistent with our study. This study revealed that after 1 month of treatment with clopidogrel bisulfate tablets combined with olmesartan medoxomil, the patients' neurological function, hemiplegic limb motor function, and activities of daily living were prominently improved. After 12 months of medication, the average neurological score of the patients recovered from severe neurological deficit to mild neurological deficit, and the motor function of most patients with hemiplegic limbs gradually recovered from paralysis and weakness to fine, stable, and coordinated movement. In addition, the modified Barthel score results showed that most patients had moderate or severe dysfunction before treatment and need help in life. After 12 months of treatment, most patients gradually recovered their ability to take care of themselves. Taken together, the combination of clopidogrel bisulfate tablets and olmesartan medoxomil had prominent clinical effects in the treatment of patients with ischemic stroke and hypertension and could remarkably improve the prognosis and improve the quality of life of patients.

A range of clinical studies confirmed that hypertension is one of the crucial risk factors for the onset and recurrence of ischemic stroke [32]. Hypertension can facilitate the disease of the patient's blood vessel wall and increase the incidence of ischemic stroke and subsequent neurodegeneration [33, 34]. To further study the prognostic factors of patients with ischemic stroke and hypertension, this study divided the patients into two groups according to the expression level of plasma AT_1_R before treatment. The results expressed that patients with high levels of plasma AT_1_R expression before treatment had a higher risk of stroke recurrence and further enlargement of cerebrovascular residual lesions within 12 months of treatment. It indicated that ischemic stroke accompanied by high plasma AT_1_R expression was closely related to the prognosis of patients. Consistent with our results, a 5-year follow-up survey of patients with a history of hypertension and stroke or transient ischemic attack uncovered that lowering blood pressure has a beneficial effect in the secondary prevention of stroke [35]. Besides, it was found that compared with other ARBs, olmesartan can more effectively reduce blood pressure in patients with a history of stroke or asymptomatic cerebral infarction [36]. As suggested by these findings, the combined treatment regimen of clopidogrel bisulfate tablets and olmesartan medoxomil was highly targeted to the treatment of patients with ischemic stroke and hypertension, and controlling blood pressure was of great significance for the treatment of patients with ischemic stroke and hypertension.

However, our results revealed that the expression level of AT_1_R had no marked effect on the mortality of patients, which may be related to the insufficient sample size, especially after being divided into high/low AT_1_R expression level groups, which was the limitation of this study. Additionally, due to the limitation of sample size, this study failed to control confounding factors (such as age and gender) for further stratification analysis, and stratification analysis would reduce the credibility of statistical analysis results. Hence, the sample size needs to be further expanded in future research.

## 5. Conclusion

Collectively, the combination of clopidogrel bisulfate tablets and olmesartan medoxomil in the treatment of ischemic stroke patients combined with hypertension can achieve satisfactory therapeutic effects, help reduce the long-term recurrence rate of stroke, and is worthy of clinical application. Moreover, AT_1_R level may be a vital factor affecting the prognosis of patients with ischemic stroke and hypertension, and it can offer new ideas for clinical diagnosis and prognostic evaluation.

## Figures and Tables

**Figure 1:** Flow chart for screening patients.

**Figure 2:** Cerebrovascular residual lesions in ischemic stroke patients with hypertension in high- and low-AT_1_R groups. Yellow represents the low-AT_1_R group, blue represents the high-AT_1_R group, and the box represents censored patients; *p* = 0.029.

**Figure 3:** Recurrence rate of ischemic stroke patients combined with hypertension in high- and low-AT_1_R groups. Yellow represents the low-AT_1_R group, blue represents the high-AT_1_R group, and the box represents censored patients; *p* = 0.016.

**Figure 4:** The overall survival rate of ischemic stroke patients with hypertension in high- and low-AT_1_R groups. Yellow represents the low-AT_1_R group, blue represents the high-AT_1_R group, and the box represents censored patients; *p* = 0.541.

**Table 1:** Clinical characteristics of patients.

Characteristic	
Age (years), average value ± SD	63.96 ± 6.10
Male, *n* (%)	52 (57.78)
Time from onset to admission (h), average value ± SD	20.33 ± 5.08
BMI, average value ± SD	24.29 ± 3.24
Smoking history, *n* (%)	32 (35.6%)
Drinking history, *n* (%)	11 (12.22%)
LDL cholesterol (mg/dL), average value ± SD	112.72 ± 12.25
Blood sugar (mg/dL), average value ± SD	125.77 ± 11.41
BUN/Cr ratio ≥ 15, *n* (%)	74 (82.22%)
Systolic blood pressure (mmHg), average value ± SD	162.02 ± 10.14
Diastolic blood pressure (mmHg), average value ± SD	93.12 ± 7.57
AT_1_R (*μ*g/L), average value ± SD	5.11 ± 0.84

**Table 2:** Comparison of MESSS scores before and after treatment.

Time	MESSS score	*t*	*p*
Before treatment	31.00 ± 5.82		
1 month	30.08 ± 5.77	2.94	0.004
2 months	23.30 ± 5.82	15.46	<0.001
3 months	16.93 ± 4.78	38.67	<0.001
6 months	10.37 ± 3.88	48.70	<0.001
9 months	8.52 ± 3.11	63.60	<0.001
12 months	7.33 ± 2.63	60.76	<0.001

**Table 3:** Comparison of Brunnstrom score before and after treatment.

Time	Brunnstrom score	*t*	*p*
Before treatment	1.83 ± 0.66		
1 month	2.07 ± 0.75	-3.30	0.001
2 months	3.28 ± 1.00	-17.93	<0.001
3 months	4.07 ± 0.83	-33.44	<0.001
6 months	4.55 ± 0.75	-52.06	<0.001
9 months	4.92 ± 0.80	-53.41	<0.001
12 months	5.15 ± 0.76	-47.28	<0.001

**Table 4:** Comparison of modified Barthel score before and after treatment.

Time	Modified Barthel score	*t*	*p*
Before treatment	41.17 ± 11.44		
1 month	44.83 ± 10.69	-4.56	<0.001
2 months	55.75 ± 11.63	-17.96	<0.001
3 months	67.62 ± 11.99	-35.30	<0.001
6 months	74.17 ± 13.37	-49.42	<0.001
9 months	79.18 ± 12.61	-65.54	<0.001
12 months	85.96 ± 10.48	-71.15	<0.001

## Data Availability

The datasets used and/or analyzed during the current study are available from the corresponding author on reasonable request.
